This article has been retracted.

# High CHAF1A Expression Levels Are Positively-Correlated with PD-L1 Expression and Indicate Poor Prognosis in Gastric Cancer

**DOI:** 10.1155/2022/1323321

**Published:** 2022-07-19

**Authors:** Zhehan Bao, Yanqiang Zhang, Pengcheng Yu, Yi Wang, Can Hu, Yuhang Xia, Li Yuan, Zhiyuan Xu, Xiangdong Cheng

**Affiliations:** ^1^The First Clinical Medical College of Zhejiang Chinese Medical University, Hangzhou 310053, China; ^2^The Cancer Hospital of the University of Chinese Academy of Sciences (Zhejiang Cancer Hospital), Institutes of Basic Medicine and Cancer (IBMC), Chinese Academy of Sciences, Hangzhou 310022, China; ^3^Zhejiang Key Lab of Prevention, Diagnosis, and Therapy of Upper Gastrointestinal Cancer, Zhejiang Cancer Hospital, Hangzhou 310022, China; ^4^Department of Chinese Surgery, Linping District Hospital of Traditional Chinese Medicine, Hangzhou 311100, China

## Abstract

**Objective:**

The aim of this study was to analyze the association between the expression of chromatin assembly factor 1 subunit A (CHAF1A) in gastric cancer (GC) and clinicopathological features, disease prognosis, and expression of programmed cell death-ligand 1 (PD-L1). *Material and Methods*. A total of 140 GC tissue specimens were collected between January 2013 and December 2017. CHAF1A expression in GC and paracancerous tissues was determined. Then, the associations between CHAF1A expression level in the collected tissues and clinicopathological features as well as PD-L1 expression level were investigated. Cox regression analyses were carried out to determine whether CHAF1A is an independent prognostic factor for GC. Finally, the association between CHAF1A expression levels and survival of the GC patients was investigated.

**Results:**

A significantly higher level of CHAF1A expression in GC tissues was found compared to that in paracancerous tissues (*p*=0.042). CHAF1A expression level in GC tissues was found to be strongly associated with family history (*p*=0.005), smoking history (*p*=0.016), T stage (*p*=0.001), tumor marker AFP (*p*=0.017), tumor marker CEA (*p*=0.027), and PD-L1 expression (*p*=0.029). CHAF1A expression was also found to be positively correlated to PD-L1 expression (*p*=0.012). Moreover, high CHAF1A expression levels were found to lead to poor prognosis (*p*=0.019). Univariate and multivariate analyses all showed that CHAF1A was an independent poorer prognostic factor for gastric cancer (*p*=0.021, HR = 1.175, 95% CI: 1.090–2.890 for univariate analyses; *p*=0.014, HR = 2.191, 95% CI:1.170–4.105 for multivariate analyses). A high level of CHAF1A expression was thus found to be an independent risk factor for GC prognosis.

**Conclusion:**

High CHAF1A expression is associated with poor GC prognosis and positively correlated to PD-L1 expression. Thus, CHAF1A expression level may be used as a novel biomarker for GC diagnosis.

## 1. Introduction

Gastric cancer (GC) is the fifth most common malignant tumor type worldwide [1, 2]. In 2020, approximately 1089,000 new cases and 769,000 deaths were caused by GC, which ranks fifth and fourth among malignant tumor types in terms of incidence rate and mortality, respectively [3]. Thus, GC is a serious health threat. GC also ranks third in terms of death rate among cancer types in China [4]. Despite advances in early diagnosis technology, accuracy of surgical procedures, and chemotherapy, GC is diagnosed mostly in the advanced stage due to difficulties in detecting early symptoms of GC. GC is more difficult to operate in the late stage, and also relapses more often with a high metastasis rate: 35–70% of patients experience cancer recurrence and metastasis within 5 years [5, 6]. Therefore, novel biomarkers for diagnosis, prognosis, and treatment of GC are urgently needed.

Chromatin assembly factor-1 (CAF-1) is a protein complex composed of p48, p60 and p150 (CHAF1A) subunits [7]. CAF-1 promotes DNA replication during nucleosome formation and participates in chromatin structure recovery following DNA repair [8–10]. CHAF1A is the core subunit of CAF-1 and participates in DNA replication, gene expression regulation, and DNA mismatch repair [10]. Uncontrolled CHAF1A expression plays a significant role in cancer development. For example, Han et al. found that CHAF1A was up-regulated in cervical cancer tissues, and CHAF1A expression was associated with the survival of cervical cancer patients [11]. Dasgupta et al. also revealed that CHAF1A was a prognostic marker for the recurrence of colorectal cancer [12]. On the other hand, the role of CHAF1A expression in GC remains insufficiently understood.

Programmed cell death-ligand 1 (PD-L1) is an important immune checkpoint protein [13]. Degradation of PD-L1 in proteasomes or lysosomes through a variety of pathways increases the effectiveness of cancer immunotherapy. Nevertheless, the relationship between expression levels of CHAF1A and PD-L1 remains unclear in GC. The aim of this study was thus to investigate the relationship between CHAF1A expression, clinicopathological features, and prognosis in GC, and thereby to provide insight for future research on the role of CHAF1A in GC.

## 2. Material and Methods

### 2.1. Recruitment of Participants

The participants in this study included 140 patients diagnosed with GC between January 2013 and December 2017 in the Affiliated Cancer Hospital of the Chinese Academy of Sciences (Zhejiang Cancer Hospital, Hangzhou, China). The patients were included according to the following criteria: (a) GC diagnosis based on a pathological assessment of surgical samples with complete medical records, (b) no antitumor treatments such as chemotherapy, radiotherapy, biotherapy, or immunotherapy prior to operation, and (c) voluntary participation. Patients who had another malignant tumor type in the last five years as well as metastasized tumors, and those who received preoperative antitumor therapy were excluded from the study. The clinical and pathological data of patients were collected, including age, gender, smoking history, drinking history, history of GC in the family, weight loss, T stage, N stage, M stage, TNM stage (which refers to the eighth edition of AJCC staging standard), Borrmann type, Lauren type, pathological type, degree of differentiation, tumor location, tumor size, tumor marker expression, and survival of patients. This study was approved by the ethics committee of Zhejiang Cancer Hospital, Hangzhou, China (ethic code: IRB-2021-431).

### 2.2. Immunohistochemistry Analysis

The GC and paracancerous tissue specimens were fixed by formalin and embedded in paraffin. Tissue slices were dewaxed, and washed with distilled water, and then the antigen was repaired. The slices were washed with PBS three times for 5 min each. Then, the sections were incubated overnight with primary antibodies (CHAF1A: 17037-1-AP; HER2: ab1662; PD-L1 : SK006) at 4°C, and then washed with PBS. After that, goat anti-rabbit IgG H & L (Biotin) (dilution ratio 1 : 1000)/goat anti-mouse IgG H & L (Biotin) (dilution ratio 1 : 500) were added to the tissue microarray. After incubation for 30 min, sections were washed with PBS. Then DAB color reagent kit was used for DAB staining and hematoxylin restaining of the nucleus. Finally, the tissue chip was dehydrated, and sealed with neutral gel. Representative images were taken using an Olympus IX71 microscope (Olympus, Tokyo, Japan).

The expression intensity of CHAF1A was evaluated using the H score system as follows: H score = (∑ ISxAP), where IS and AP indicates staining intensity and the percentage of positively stained cells, respectively. IS is a measure of cell staining: 0 points indicate no staining, whereas 1, 2, and 3 points indicate weak, moderate, and strong staining, respectively. The percentage levels in the range of 1–25% AP stained cells correspond to 1 point; whereas 26–50%, 51–75%, and 76–100% correspond to 2, 3, and 4 points, respectively. An H score above 1 indicated the existence of CHAF1A expression, whereas H scores below and equal to or above 6 indicated low and high CHAF1A expression levels, respectively.

IHC is the recommended method for HER2-based detection of GC according to the 2016 edition of HER2 detection guidelines for GC. Patients with IHC 3+ were considered HER2-positive, whereas patients with IHC 1+ and IHC 0 were considered HER2-negative. Cases with IHC 2+ were considered “uncertain”, for which in situ hybridization is required to confirm the HER2 status. Amplified represents HER2 positive, conversely, it means HER2 negative.

The PD-L1 expression level was corresponded to the combined positive score (CPS) score, CPS = [PD-L1 positive cells (tumor cells, lymphocytes, macrophages)/total tumor cells] *∗* 100. CPS scores higher than 10 indicated positive PD-L1 expression [14, 15].

### 2.3. Follow-Up of Participants

The follow-up of participants was mainly conducted by outpatient review and telephone interviews. The date of the last follow-up was December 2020. Overall survival (OS) refers to the time from radical surgery to death or follow-up endpoint.

### 2.4. Statistical Analysis

Measured data are expressed as median + upper and lower quartiles, whereas counted data are expressed as value and percentage, and analyzed using the chi-square test and Fisher exact test. Kaplan–Meier method was utilized for survival analysis. SPSS 26.0 and Graphpad Prism 9 were used for statistical analyses. *p* < 0.05 was considered statistically significant.

## 3. Results

### 3.1. Characteristics of Participants

A summary of the characteristic of participants is given in Table 1. A total of 140 GC patients with a median age of 61 (28, 86) years participated in this study, including 102 males (72.86%) and 38 females (27.14%). A total of 21 (15%) had a family history of GC. Furthermore, 50 (35.71%) and 34 (24.29%) patients had smoking and drinking histories, respectively. A total of 71 patients (50.71%) had moderately/highly differentiated tumors, whereas 63 patients (45%) had poorly differentiated/undifferentiated tumors, and tumor differentiation was unknown for 6 patients (4.29%). A total of 123 (87.86%), 5 (3.57%), and 12 (8.57%) patients had adenocarcinoma, signet ring cell carcinoma, and mucinous adenocarcinoma, respectively. According to the staging criteria of GC, as stated in the eighth edition of AJCC Cancer Staging Manual, 1 (0.71%), 18 (12.86%), 108 (75%), and 13 cases (9.29%) were in stages I, II, III, and IV, respectively.

### 3.2. The Association between CHAF1A Expression and Clinicopathological Features in GC

High level of CHAF1A expression was detected in 79 (56.43%) and 62 (43.57%) cases in GC and paracancerous tissues, respectively (Table 2). CHAF1A expression in GC tissues was found to be significant higher than that in paracancerous tissues (*p*=0.042) (Table 2 and Figure 1). CHAF1A expression was also found to be strongly associated with family history of GC (*χ*^2^ = 7.826, *p*=0.005), smoking history (*χ*^2^ = 5.826, *p*=0.016), T stage (*χ*^2^ = 10.989, *p*=0.001), tumor marker CEA (*χ*^2^ = 4.870, *p*=0.027), tumor marker AFP (*χ*^2^ = 5.672, *p*=0.017), and PD-L1 expression (*χ*^2^ = 4.776, *p*=0.029) (Table 3).

### 3.3. CHAF1A Expression in GC Was Not Correlated with HER2 Expression, yet Positively Correlated with PD-L1 Expression

HER2 is the first target used successfully for GC treatment and remains the most effective target to date [16]. The use of PD-1/L1 antibody in advanced GC treatment has also shown unprecedented success [17]. Thus, the relationships between CHAF1A expression, HER2, and PD-L1 expression in GC tissues, as well as the value of CHAF1A as a diagnostic and therapeutic target for GC were further evaluated. As shown in Table 4, the HER2-positive rate in GC was 12.86%, whereas the PD-L1-positive rate was 34.29%. In addition, no association was found between CHAF1A and HER2 expression levels, yet CHAF1A expression was found to be positively correlated to PD-L1 expression (Figure 2). The expression level of CHAF1A in PD-L1-positive cases was 56.25%, and that in PD-L1-negative cases was only 36.97%. There were 27 PD-L1-positive cases (19.29%) with high expression of CHAF1A, 21 PD-L1-positive cases (15%) with no CHAF1A expression, 34 PD-L1-negative cases (24.29%) with high expression of CHAF1A, and finally 92 PD-L1-negative cases (65.71%) with low expression of CHAF1A.

### 3.4. CHAF1A Is an Independent Risk Factor in GC

As shown in Figure 3(a), high CHAF1A expression was found to be associated with poor prognosis when compared to low CHAF1A expression (43.04% vs. 55.74%, *p*=0.019). In addition, univariate [HR (95% CI): 1.175 (1.090–2.890), *p*=0.021] and multivariate Cox regression analysis [HR (95% CI): 2.191 (1.170–4.105), *p*=0.014] revealed that the CHAF1A was an independent risk factor for GC patients (Tables 5 and 6). Kaplan–Meier analysis was also performed on expressions of HER2 and PD-L1. The 5-year survival rate of GC patients (Figures 3(b) and 3(c)), and HER2 and PD-L1 expression levels showed no significant effect on the prognosis of GC patients. However, when CHAF1A was included in the analysis, opposite results were observed (*p* < 0.05; Figures 3(d) and 3(e)).

## 4. Discussion

The role of CHAF1A in tumor development has been revealed in previous studies. Xia et al. found that CHAF1A up-regulation hinders cell apoptosis in epithelial ovarian cancer [18]. Wu et al. revealed that CHAF1A is a poor prognostic factor in colon cancer, and its overexpression promotes cell proliferation [19]. Cai et al. found that miR-520b hinders nonsmall cell lung cancer metastasis and proliferation by targeting CHAF1A [20]. Shen et al. also demonstrated that CHAF1A overexpression facilitates cell proliferation, and inhibits apoptosis in human retinoblastoma cells [21]. Tao et al. found that CHAF1A facilitates neuroblastoma oncogenesis and blocks neuronal differentiation through metabolic reprogramming [22]. Moreover, high levels of CHAF1A expression was found in GC tissue and cell lines, and the up-regulation of CHAF1A was found to be associated with poor clinical outcome [23]. Zheng et al. found that CHAF1A interacts with TCF4 to facilitate GC by leading to overexpression of c-MYC and CCND1 [24]. The large sample size of this study further increases the reliability of the obtained results. Kaplan–Meier analysis yielded that high CHAF1A expression level caused poor prognosis, and was an independent risk factor for GC patients, which is in line with the findings of the above studies. Moreover, CHAF1A expression levels were found to be high in patients with a family history of GC, smoking history, and later T stage. The high expression level of CHAF1A was also positively associated with tumor marker CEA, tumor marker AFP and PD-L1 expression, which supports the results of survival analysis. Taken together, our results indicate that CHAF1A has an oncogenic role in GC, and may be considered a new therapeutic target in GC.

PD-L1 suppresses T cell activation and leads to tumor progression. Wei et al. found that PD-L1 facilitates the expansion of colorectal cancer stem cells by activating HMGA1-dependent signaling pathways [25]. Zhang et al. discovered an association between PD-L1 expression and shorter OS in GC patients [26]. PD-L1 is also a predictive immune checkpoint inhibitor therapy marker [27]. PD-L1 plays the role of a “brake” in immune function, and immune checkpoint inhibition is effective in reactivating T cells and eliminating cancer cells [28]. Anti-PD-L1/PD-1 antibodies are also very useful for the treatment of GC [29]. Kang et al. found that nivolumab, another humanized IgG4 recombinant anti-PD-1 monoclonal antibody, significantly prolonged OS in patients with advanced GC as a third-line therapy [30]. Here, CHAF1A expression was not found to be associated with the expression of HER2 expression, yet positively associated with PD-L1 expression. Moreover, HER2 and PD-L1 had no significant effect on the prognosis of GC patients. However, when CHAF1A was included, opposite results were obtained, which indicate that CHAF1A may be a potential target to improve the therapeutic effectiveness of PD-L1 inhibitors in GC.

On the other hand, this study also has several limitations. First, more clinicopathological features should be included to explore the associations between CHAF1A expression and clinicopathological features. Second, the molecular mechanism underlying the positive association between CHAF1A expression and PD-L1 expression should be clarified.

## 5. Conclusions

CHAF1A is highly expressed in GC tissues, and this high level of expression indicates a poor prognosis. CHAF1A expression is also closely related to the family history of GC, smoking history, T stage, tumor marker CEA, tumor marker AFP and PD-L1 expression. Finally, CHAF1A expression is also positively correlated to PD-L1 expression.

## Figures and Tables

**Figure 1:** Chromatin assembly factor 1 subunit A (CHAF1A) is upregulated in gastric cancer (GC) tissues. (a) CHAF1A expression statistics in GC and paracancerous tissues. (b) representative images of CHAF1A expression in GC and paracancerous tissues (200x).

**Figure 2:** Programmed cell death-ligand 1 (PD-L1) is upregulated in gastric cancer (GC) tissue. (a) PD-L1 expression statistics in GC tumor tissues. (b) HER2 expression statistics in GC tumor tissues. (c) Representative images of PD-L1 and HER2 expression in GC and paracancerous tissues (200x).

**Figure 3:** The Kaplan–Meier survival analysis shows an association between the expression of chromatin assembly factor 1 subunit A (CHAF1A), programmed cell death-ligand 1 (PD-L1), HER2 expression, and GC prognosis. (a) The survival curve shows that the 5-year overall survival (OS) of patients with high CHAF1A expression is significantly lower than that of patients with low CHAF1A expression (43.04% vs 55.74%, *p*=0.019). (b) Kaplan–Meier survival analysis of PD-L1. (c) Kaplan–Meier survival analysis of HER2. (d) Kaplan–Meier survival analysis of CHAF1A combined with PD-L1. (e) Kaplan–Meier survival analysis of CHAF1A combined with HER2.

**Table 1:** Participants characteristic.

Clinicopathological features	Number (%)
Age (year)	61 (28,86)

Gender	
Male	102 (72.9%)
Female	38 (27.1%)

Family history (gastric cancer)	
Yes	21 (15%)
No	119 (85%)

Smoking history	
Yes	50 (35.7%)
No	90 (64.3%)

Drinking history	
Yes	35 (25%)
No	105 (75%)

Weight lose	
Yes	53 (37.9)
No	87 (62.1%)

Tumor location	
Proximal	47 (33.6%)
Distal	86 (61.4%)
Unknown	7 (5%)

Borrmann type	
I	3 (2.1%)
II	76 (54.3%)
III	43 (30.7%)
IV	16 (11.4%)
Unknown	2 (1.4%)

Lauren type	
Intestinal	67 (47.9%)
Diffuse	51 (21.4%)
Mixed	21 (15%)
Unknown	1 (0.7%)

Tumor size (cm)	
≥ 5	89 (63.6%)
< 5	50 (35.7%)
Unknown	1 (0.7%)

Grade of differentiation	
Poor	63 (45%)
Moderate-poor	49 (35%)
Moderate	21 (15%)
Well	1 (0.7%)
Unknown	6 (4.3%)

Pathological type	
Adenocarcinoma	123 (87.9%)
Mucinous adenocarcinoma	12 (8.6%)
Signet ring cell carcinoma	5 (3.6%)

T stage	
1	2 (1.4%)
2	6 (4.3%)
3	13 (9.3%)
4	119 (85%)

N stage	
0	11 (7.9%)
1	31 (22.1%)
2	38 (27.1%)
3	60 (42.9%)

M Stage	
0	127 (90.7%)
1	13 (9.3%)

TNM stage	
I	1 (0.7%)
II	18 (12.9%)
III	108 (77.1%)
IV	13 (9.3%)

AFP (ng/ml)	
≤ 8.1	131 (93.6%)
> 8.1	7 (5%)
Unknown	2 (1.4%)

CEA (ng/ml)	
≤ 5	102 (72.9%)
> 5	38 (27.1%)

CA199 (U/ml)	
≤ 37	96 (68.6%)
> 37	44 (31.4%)

CA724 (U/ml)	
≤ 6.9	92 (65.7%)
> 6.9	32 (22.9%)
Unknown	6 (4.3%)

CA125 (U/ml)	
≤ 35	129 (92.1%)
> 35	11 (7.9%)

CA50 (U/ml)	
≤ 25	68 (48.57%)
> 25	19 (13.57%)
Unknown	53 (37.86%)

**Table 2:** CHAF1A expression in gastric cancer and paracancerous tissues.

Variables	*N*	CHAF1A expression			*χ* ^2^	*p*-value
		High	Low	High rate		
Tumor tissue	140	79	61	56.43%	4.129	**0.042** ^*∗*^
Paracancerous tissue	140	62	78	44.29%		

^*∗*^Statistically significant (*p* < 0.05).

**Table 3:** The correlations between the CHAF1A expression levels and the clinicopathological features of gastric cancer patients and the univariate analysis of gastric cancer patients.

Variables	CHAF1A expression		Total	High rate	*χ* ^2^	*p*-value
	High	Low				
Age (years)						
≤ 60	56	27	83	67.47%	3.140	0.076
＞ 60	30	27	57	52.63%		

Gender						
Male	62	40	102	60.78%	2.290	0.089
Female	17	21	38	44.74%		

Family history (gastric cancer)						
Yes	17	4	21	80.95%	7.826	**0.005** ^*∗*^
No	57	62	119	47.90%		

Smoking history						
Yes	35	15	50	70%	5.826	**0.016** ^*∗*^
No	44	46	90	48.89%		

Drinking history						
Yes	16	19	35	45.71%	0.087	0.768
No	45	60	105	42.86%		

Weight loss						
Yes	30	23	53	56.60%	0.001	0.794
No	49	38	87	56.32%		

Tumor location						
Proximal	34	13	47	72.34%	0.001	0.425
Distal	42	44	86	48.84%		
Unknown	3	4	7	42.86%		

Borrmann type						
I/II	46	33	79	58.23%	0.679	0.410
III/IV	33	26	59	55.93%		
Unknown	0	2	2	0		

Lauren type						
Intestinal	41	26	67	61.20%	1.232	0.540
Mixed	12	9	21	57.14%		
Diffuse	26	25	51	50.98%		
Unknown	0	1	1	0		

Tumor size (cm)						
> 5 cm	52	37	89	58.42%	0.257	0.613
≤ 5 cm	27	23	50	54%		
Unknown	0	1	1	0		

Grade of differentiation						
Poor/moderate-poor	31	32	63	49.21%	2.207	0.137
Moderate/well	44	27	71	61.97%		
Unknown	4	2	6	66.67%		

T stage						

T1/2	0	8	8	0%	10.989	**0.001** ^*∗*^

T3/4	79	53	132	59.85%		

N stage						
N0/1	26	16	42	61.90%	0.732	0.392
N2/3	53	45	98	54.08%		

M stage						
M0	70	57	127	55.12%	0.955	0.328
M1	9	4	13	69.23%		

TNM stage						
Ι/II	8	11	19	42.11%	1.635	0.201
III/IV	71	50	121	58.68%		

HER-2						
Positive	5	13	18	27.78%	2.096	0.148
Negative	56	66	122	45.90%		

PD-L1						
Positive	27	21	48	56.25%	4.776	**0.029** ^*∗*^
Negative	34	58	92	36.96%		

AFP (ng/ml)						
≤ 8.1	71	60	131	54.20%	5.672	**0.017** ^*∗*^
＞ 8.1	7	0	7	100%		
Unknown	1	1	2	50%		

CEA (ng/ml)						
≤ 5	52	50	102	50.98%	4.870	**0.027** ^*∗*^
＞ 5	27	11	38	71.05%		

CA199 (U/ml)						
≤ 37	52	44	96	54.17%	0.050	0.824
＞ 37	27	17	44	61.36%		

CA724 (U/ml)						
≤ 6.9	41	51	92	44.57%	0.051	0.821
＞ 6.9	15	17	32	46.88%		
Unknown	5	11	16	45.45%		

CA125 (U/ml)						
≤ 35	70	59	129	54.26%	0.309	0.578
＞ 35	7	4	11	63.64%		

CA50 (U/ml)						
≤ 25	33	35	68	48.53%	0.459	0.498
＞ 25	6	4	19	60.0%		
Unknown	20	33	53	37.73%		

^*∗*^Statistically significant (*p* < 0.05).

**Table 4:** Differential expression of HER-2 and PD-L1.

Variables	*N*	CHAF1A expression		
		Negative	Positive	High rate (%)
HER-2	140	122	18	12.86
PD-L1	140	92	48	34.29

^*∗*^Statistically significant (*p* < 0.05).

**Table 5:** Univariate cox regression analysis of 140 gastric cancer patients.

Parameters	Univariate analysis	
	*p* value	HR (95% CI)
Gender		
Female vs. male	0.836	1.082 (0.513–2.279)

Age (year)		
≤ 65 vs. ＞ 65	0.651	1.168 (0.595–2.295)

CHAF1A expression		
Low vs. high	**0.021** ^*∗*^	1.175 (1.090–2.890)

Gastric history		
No vs. yes	0.053	2.719 (0.988–7.487)

Smoking history		
No vs. yes	0.920	1.036 (0.519–2.070)

Drinking history		
No vs. yes	0.848	0.927 (0.428–2.008)

Weight loss		
No vs. yes	0.340	1.398 (0.703–2.788)

Tumor location		
Proximal	0.662	
Distal		
Total		

Borrmann type		
I, II vs. III, IV	**0.003** ^*∗*^	2.864 (1.420–5.777）

Lauren type		
Intestinal	0.382	
Diffuse		
Mixed		

Tumor size (cm)		
≤ 5 vs. ＞ 5	0.258	1.491 (0.747–2.979)
Grade of differentiation poor/moderate-poor.vs.moderate/well	0.398	1.341 (0.679–2.647)

T sstage		
T1,T2 vs.T3,T4	0.144	3.387 (0.659–17.398)

N stage		
N0,N1 vs.N2,3	**0.001** ^*∗*^	3.947 (1.804–8.638)

M stage		
M0 vs.M1	**0.014** ^*∗*^	13.400 (1.692–106.142)

TNM stage		
I,II vs. III,IV	0.177	1.990 (0.733–5.400)

Pathological type		
Adenocarcinoma with others	0.201	1.904 (0.696–5.207)

AFP (ng/ml)		
≤ 8.1 vs.＞ 8.1	0.308	2.388 (0.447–12.752）

CEA (ng/ml)		
≤ 5 vs.＞ 5	**0.006** ^*∗*^	3.109 (1.393–6.938)

CA199 (U/ml)		
≤ 37 vs.＞ 37	**0.045** ^*∗*^	1.589 (1.011–2.496）

CA125 (U/ml)		
≤ 35 vs. ＞ 35	**0.025** ^*∗*^	10.806 (1.344–86.885)

CA50		
≤ 25 vs. ＞ 25	0.165	2.204 (0.723–6.728)

PD-L1		
Negative vs. positive	0.777	1.106 (0.552–2.217)

HER-2		
Negative vs. positive	0.517	1.406 (0.503–3.391)

^*∗*^Statistically significant (*p* < 0.05).

**Table 6:** Multivariate cox regression analysis of 140 gastric cancer patients.

Factors	*B*-value	Multivariate analysis			
		SE	Wald	*p*	HR (95% CI)
Sex					
Male vs.female	0.59	0.393	2.257	0.133	1.804 (0.835–3.897)

Age (year)					
≤ 60 vs.＞ 60	−0.179	0.297	0.363	0.547	0.836 (0.468–1.496)

CHAF1A expression					
High vs. low	0.784	0.32	5.998	**0.014** ^*∗*^	2.191 (1.170–4.105)

Family history (GC)					
Yes vs. no	1.077	0.396	7.405	**0.007** ^*∗*^	2.936 (1.352–6.377)

Smoking					
Yes vs.no	−0.609	0.356	2.919	0.088	0.544 (0.271–1.094)

Drinking					
Yes vs. no	0.254	0.372	0.464	0.496	1.289 (0.621–2.674)

Weight loss					
Yes vs. no	0.007	0.310	0.000	0.983	1.007 (0.548–1.849)

Tumor location				0.164	
Distal vs. proximal	0.427	0.353	1.465	0.226	1.533 (0.767–3.064)
Total vs. proximal	1.146	0.641	3.196	0.074	3.145 (0.895–11.044)

Borrmann type					
I,IIvs.III,IV	0.831	0.327	6.45	**0.011** ^*∗*^	2.295 (1.209–4.356)

Lauran type				0.712	
Mixed vs. Intestinal	−0.266	0.332	0.638	0.424	0.767(0.400–1.471)
Diffuse vs. Intestinal	−0.039	0.452	0.008	0.931	0.961 (0.396–2.333)

Tumor size					
≤ 5 cm vs.＞ 5 cm	−0.178	0.337	0.279	0.597	0.837 (0.433–1.619)

Pathological type					
Adenocarcinoma vs. others	0.763	0.422	3.272	0.07	2.144 (0.938–4.900)

TNM stage					
I,II vs. III,IV	−0.071	0.466	0.023	0.879	0.931 (0.374–2.322)

AFP (ng/ml)					
≤ 8.1 vs.＞ 8.1	0.171	0.591	0.084	0.772	1.187 (0.373–3.777)

CA199 (U/ml)					
≤ 37 vs.＞ 37	0.254	0.329	0.595	0.44	1.289 (0.676–2.459)

CA125 (U/ml)					
≤ 35 vs. ＞ 35	1.079	0.464	5.392	**0.02** ^*∗*^	2.941 (1.183–7.308)

HER2					
Negative vs.positive	0.093	0.436	0.045	0.831	1.098 (0.467–2.582)

PD-L1					
Negative vs.positive	0.096	0.296	0.105	0.746	1.101 (0.616–1.968)

^*∗*^Statistically significant (*p* < 0.05).

## Data Availability

All data generated or analyzed during this study are included within this article.

## Additional Points

(1) High CHAF1A expression is associated with poor gastric cancer prognosis. (2) CHAF1A expression was positively correlated with PD-L1 expression in gastric cancer. (3) CHAF1A is an independent prognostic factor in GC.
